The article "Street Landscape Planning and Design Guided by Artificial Intelligence Interactive Experience" was retracted in 2023. Reasons: unreliable results or conclusions; concerns about the data; concerns about the peer review; concerns about the citations.

# Street Landscape Planning and Design Guided by Artificial Intelligence Interactive Experience

**DOI:** 10.1155/2022/3146637

**Published:** 2022-08-23

**Authors:** Jun Xie, Dandan Wang

**Affiliations:** College of Architecture and Civil Engineering, Qiqihar University, Qiqihar, Heilongjiang 161006, China

## Abstract

As an important part of the city, urban streets have always played an active role in carrying public needs and optimizing public living spaces. They are also important to open public spaces in the city. In addition, with technology integration and life, the interactive experience of artificial intelligence (AI) in Street View is gradually increasing. A streetscape planning and design method based on AI interactive experience is proposed. CSiXRevit 2022 software builds street simulation models for better street planning and design. Street digital imaging technology is used to analyze the original streetscape. Landscape features are integrated with the street model. Based on intelligent technology, urban landscape design is studied, and AI interactive experience is analyzed. Analytic hierarchy process (AHP) and AI technology evaluate the effect of landscape design. Firstly, AHP is used to construct the evaluation index system of the rural landscape design effect, and the index weight is determined. Back propagation neural network (BPNN) is used to construct an evaluation model of landscape design effect. Three indexes of target, project, and indicator layer are used to evaluate the effect of rural landscape design. The results show that (1) the variety and richness of streetscapes in the survey area should be increased. Interactive buildings should be placed on the street. (2) The comprehensive evaluation score of the street landscape is 0.60, and the design effect is excellent. The comprehensive evaluation values of the three project layers are 0.65, 0.48, and 0.67, respectively. The data show that the carrying capacity index of the study area is the best, and the vitality index is the weakest. Therefore, when designing the street landscape, the economic development has been strengthened by attracting investment, introducing large-scale exhibition shops, increasing street income, strengthening the construction of street public facilities, and paying attention to the public street experience. This work can provide references for related streetscape designs.

## 1. Introduction

Good services and products have been unable to meet the needs of people's spiritual civilization fully. Therefore, the advent of the economic era creates value for emotional needs. Streets are created with the formation of cities. It is formed by the road as the carrier, has the function of passing, and is a linear space [1]. The street is a space enclosed by the building faces on both sides. The building envelope on both sides and the pavement with traffic function together form the street space. The street is an important activity place for urban residents, and it is an urban belt-shaped living space integrating cultural display, leisure and entertainment, and transportation [2]. The content of the street space is relatively rich, which can be understood as a collection that accommodates people, buildings, street furniture, and green street vegetation. As a “linear” space, it is a form of the spatial organization of human social life [3]. People's requirements for the quality of life are getting higher and higher. The improvement of science and technology and changes in people's lifestyles have led to the diversification of outdoor activities. This requires that landscape design is superficial and pays more attention to practicality [4]. Most of the current traditional landscape design methods are designed by the designer's team, with the designer's own perspective as the main design direction, and lack of in-depth research on users [5], including behavior, psychology, age, and ability. Secondly, designers lack a sense of self-substitution. Ultimately, the design is less about the experience and more about landscaping. The different needs of different groups of people are difficult to take care fully. The interactive experience with the landscape and the environment is also lacking [6, 7]. Human understanding of AI continues to deepen. Smart technology is also gradually integrated into all aspects of life. Roberts observed that recreational activities in British towns and urban centers continued to expand and analyzed other reasons why landscape design creative areas have become desolate and uninhabited areas in the context of landscape economy [8]. Anne compared the relationship between landscape design lighting color and people's night economic behavior [9]. Yeo and Heng analyzed landscape design from the perspective of sociology. They pointed out that Singapore's night landscape not only is conducive to activating the economic vitality of the society but also contributes to the sustainable development of the society [10]. At present, streetscape designers should fully use modern concepts, coordinate functional and aesthetic needs, and design streetscape schemes with the help of AI technology [11]. Intelligent public facilities and Street View systems can not only achieve the goal of resource sharing but also promote local cultural customs and appropriately relieve the psychological pressure of surrounding people [12]. In recent years, AI technology has developed rapidly as an emerging technology. At present, the widespread application of this technology improves people's lives. AI optimization technology is applied in intelligent streetscape design, which can effectively promote the good development of intelligent buildings. The new intelligent form of mechanical construction can promote the development of intelligent streetscape design and improve the application value of AI optimization technology.

At present, most of the research on interaction design focuses on industrial design and the Internet industry and has achieved remarkable results. When people analyze the interaction behavior, the interaction is regarded as the product of the public and people, reflected in the interaction process between people and the interface. People are the center of the interactive behavior of streetscape space, and the evaluation must be people-centered. Therefore, whether the interaction design is beneficial to human interests is the main evaluation criterion [13]. The AI interactive experience guides them. This work plans and designs urban streetscapes. AHP and AI techniques are used to evaluate the effectiveness of urban streetscape designs. Firstly, AI technology is analyzed and researched, and appropriate AI technology is selected according to the results. Then, the relevant software equipment and image analysis methods are described. The satisfaction of street landscape design is investigated according to AHP and back propagation neural network (BPNN) technology to judge the design effect. The innovation lies in paying more attention to the user's AI interactive experience based on traditional street landscape design and innovatively constructing a new street landscape design model based on intelligent technology. Additionally, the BPNN algorithm can improve the reliability of the experimental results by analyzing the data.

## 2. Methods

### 2.1. Interaction Analysis of AI

Intelligent interaction technology (human-computer interaction technology) is a comprehensive subject that studies the interaction between humans and computers, involving computer science, psychology, sociology, ergonomics, and other research fields. Human-computer interaction (HCI) technology refers to the technology that realizes human-computer dialogue effectively through computer input and output devices and studies how to realize multi-mode intelligent information interaction between humans and machines through vision, smell, hearing, and touch [14]. The realization of HCI technology depends on the exploration of human cognition. The development of human intelligence goes through a super-circular process in which the existing cognitive structure and the unknown cognitive structure interact and become cause and effect. The human brain acquires cognition of external things through continuous learning, perception, memory, thinking, and other physiological activities [15]. This cognitive hypercycle process can be understood as a cognitive model; that is, through the fusion of sensor information, the recognition and understanding of the target are realized. Each sensor is controlled according to the existing knowledge [16].

Inseparable from the intelligent interaction technology is the HCI interface. Interaction means a description of the relationship or state between humans and machines. Interface refers to the specific expression between human and machine, that is, the user-visible part of HCI, such as a touch-screen display [17]. Street View intelligent interaction design focuses on HCI, which interfaces can best help improve the quality of the landscape or solve difficult problems in the design [18]. Additionally, intelligent interaction intersects with the three disciplines of digital technology, AI, and interaction design. They are also inseparable, forming a common development trend of mutual dependence and progress [19]. The relationship between intelligent interaction and digital technology, AI, and interaction design is shown in Figure 1.

In Figure 1, the core of digital technology is computer technology. The classification of computer technology disciplines can be divided into interaction design, intelligent interaction, and AI. The realization of intelligent interactive technology depends on digital technology. Digital technology converts external information into binary digital data and then uses a computer to process binary data and make feedback to realize the interaction between computer and human [20]. AI is a branch of computer science. This technology attempts to understand the nature of intelligence. It wants to create a new type of intelligent machine that responds similarly to human intelligence. Its essence is to simulate the human thinking process. Machines or equipment based on intelligent interactive technology cannot replace humans. AI focuses on technology, that is, how to make machines think, work, communicate, and make decisions like human beings, and finally complete high-intensity and low-difficulty tasks instead of human beings [21]. Intelligent interaction and interaction design are two comprehensive disciplines. Usually, both intelligent interaction and interaction design originate from computer science. In contrast, interaction design is split from the field of intelligent interaction and becomes a sub-concept under the concept of intelligent interaction. Although the research focuses of the two disciplines are different, they share a common research object—people [22]. In fact, as a kind of artificial system, the ultimate purpose of a computer system is to help human beings and help one or more people outside the system. Therefore, intelligent interaction and interaction design are indistinguishable but have different emphases from each other.

The development process of AI technology can be divided into six stages. (1) The initial development period: After the concept of AI is proposed, several eye-catching results have been successfully achieved, such as machine theorem proving and checkers programs. (2) Reflect on the development period: Breakthroughs in the early stages of AI's development have greatly increased expectations for AI. People have begun to try more challenging tasks and put forward some unrealistic research and development (R&D) goals. However, failures and the failure of expected goals (e.g., the inability to use machines to prove that the sum of two continuous functions is a continuous function, machine translation errors, etc.) have brought the development of AI to a low point. (3) Application development period: The expert system in the 1970s simulates the knowledge and experience of human experts to solve problems in specific fields and realizes a breakthrough in AI from theory to practical application, from general reasoning strategy discussion to the use of specialized knowledge. Expert systems have succeeded in medicine, chemistry, and geology, pushing AI into a new climax of application development [23]. (4) Downturn development period: As the application scale of AI continues to expand, the problems of expert systems include narrow application fields, lack of commonsense knowledge, difficulty in acquiring knowledge, single reasoning method, lack of distributed functions, and difficulty in compatibility with existing databases gradually exposed [24]. (5) Steady development period: The development of network technology, especially Internet technology, has accelerated the innovation and research of AI and promoted the further practical application of AI technology. In 1997, the International Business Machines Corporation (IBM) Deep Blue computer defeated world chess champion Garry Kasparov (Russian: Гарри Каспаров). In 2008, IBM proposed the concept of a “Smarter Planet.” (6) A period of vigorous development: Computing platforms such as ubiquitous perception data and graphics processors have promoted the rapid development of AI technology represented by deep neural networks, which has greatly crossed the gap between science and application. The “technical barrier” includes image classification, speech recognition, knowledge quiz, man-machine game, driverless, and other AI technologies. These technologies have achieved technological breakthroughs from “unusable” to “useable,” ushering in a new climax of explosive growth. At this time, AI technology has developed more maturely than earlier technologies and can better improve work efficiency and handle daily affairs [25].

The streetscape design guided by the new intelligent interactive experience is different from the traditional streetscape design. It not only is a unilateral landscape theme but also considers people's experiences in the street. The main objects of the landscape design of the intelligent interactive experience street are shown in Figure 2.

In Figure 2, the main design body of the intelligent interactive experience landscape mainly has two parts. The first part is people, that is, tourists or visitors who visit the landscape area. The second part is machines, equipment, or systems, that is, the carrier of intelligent interaction. The thinking that traditional landscape design can bring to people is limited. Whether it is a figurative or abstract landscape intentional design, the landscape cannot more actively feed back people's “real emotions.” If the landscape can give some responses in terms of sound, light, shape, color, etc., through the addition of intelligence, then visitors will get obvious responses and are willing to think constantly. Additionally, through these changes, more people are attracted to participate in the interaction. Therefore, the design of the main body of the intelligent interactive landscape becomes particularly important. The carrying subject should not only be integrated into the landscape but also stand out from the surrounding landscape so that visitors can actively interact and think [26].

### 2.2. Image Analysis Technology

Digital image processing refers to converting image signals into digital signals and processing them with a computer. Image processing first appeared in the 1950s. At that time, electronic computers had developed to a certain level, and people began to use computers to process graphics and information. Digital image processing as a discipline was formed around the early 1960s. Early image processing was to improve the quality of images, taking people as objects and improving the visual effects of people—image processing input images with low quality and output images with improved quality. Image processing methods include enhancement, restoration, coding, compression, and so on. Common methods of digital image analysis technology include transformation, coding, compression, enhancement and restoration, segmentation, description, and classification. According to the characteristics of the streetscape design model, neural network image classification techniques are used to identify streetscape images.

Firstly, the neural network image classification algorithm uses principal component analysis (PCA) technology to extract the samples and the feature codes of the images to be classified. Then, the feature code is fed into the neural network for training, and the image of the unknown category is fed into the neural network to identify its type automatically. (1) PCA technology is used to extract the image feature code of each sample. (2) The sample feature code generates the input item. The category to which the sample belongs generates the corresponding output item. (3) The input and output items are sent to the nonlinear neural network for training. (4) PCA technology generates the feature code of the image to be classified. (5) The feature code of the image to be classified is sent to the neural network simulation test, and the category to which it belongs is determined according to the output item of the neural network.

### 2.3. Analytic Hierarchy Process

AHP combines qualitative and quantitative, systematic, hierarchical analysis methods. It is characterized by an in-depth study of the nature, influencing factors, and internal relations of complex decision-making problems. The thinking process of decision-making is abstracted by using less quantitative information, which is multi-objective, multi-criteria, or no-nonsense decision-making. Complex decision-making problems with structural characteristics provide easy decision-making methods. The principle of AHP is to decompose the problem into different components according to its nature. The overall goal is achieved. The interaction and subordination of each factor are combined and aggregated at different levels to form a multi-level analytical structure model. The problem is boiled down to the relative importance or merit of the order of values of the lowest level (used to make decisions about options, measures, etc.) versus the highest level (overall goals) of the program. AHP mainly includes four steps, as shown in Figure 3.

In Figure 3, the basic steps of the analytic hierarchy process include (1) the establishment of a hierarchical structure model. The decision objectives, factors (decision criteria), and objects are divided into the highest, middle, and lowest levels according to their mutual relations, and the hierarchical structure chart is drawn. The highest level (target) mainly refers to the purpose of decision-making and solving the problem. The middle layer (criteria layer or index) refers to the factors and decision-making criteria to be considered when conducting AHP. The lowest level (scheme) is the alternative at decision time. (2) Construct a judgment (pairwise comparison) matrix. The pairwise comparison matrix compares the relative importance of all factors in this layer to a certain factor in the previous layer. (3) Hierarchical ordering and consistency check: The weights of the relative importance of a factor at the same level and the next level are sorted. This process is called single-level ranking. Consistency testing determines the allowable range of inconsistency between pairwise comparison matrices. The consistency index is shown in

(1) $$\begin{array}{c} CI=\frac{\left(\lambda -n\right)}{\left(n-1\right)}. \end{array}$$

*λ* is the largest eigenvalue; *n* is the eigenvector corresponding to the eigenvalue; CI is the consistency index value. When CI = 0, the model has complete consistency; when CI is close to 0, there is satisfactory consistency; the larger the CI, the more serious the inconsistency. A random consistency index RI is introduced to measure the size of CI, as shown in

(2) $$\begin{array}{c} RI=\frac{CI1+CI2+\ldots CI500}{500}\\ =\frac{\lambda 1+\lambda 2+\ldots +\lambda 500}{\left(n-1\right)}-n. \end{array}$$

The definition of the consistency ratio is shown in

(3) $$\begin{array}{c} CR=\frac{CI}{RI}. \end{array}$$

(4) Hierarchies are sorted, and consistency is checked. Calculating the relative importance of all factors of a certain level to the highest (total target) is called the total ranking. This process is carried out sequentially from the highest to the lowest level. Additionally, the total order consistency ratio of the data is calculated.

### 2.4. Technical Analysis of BPNN

BPNN, with learning rules as the core, is a machine learning algorithm of AI technology. Forward and back propagation are two parts formed. BPNN can learn and store many input-output pattern mapping relationships without revealing the mathematical equations describing this mapping relationship in advance. Its learning rule is to use the steepest descent method. Back propagation is used to continuously adjust the weights and thresholds of the network to minimize the sum of squared errors. The topology of the BPNN model includes input, hidden, and output layers. The structure and learning operation steps of BPNN are shown in Figure 4.

In Figure 4(a), the classic BPNN contains three layers. Red represents the input layer, green represents the hidden layer, and purple represents the output layer. When a neural network is designed, the number of nodes in the input and output layer is often fixed. The middle layer can be freely specified. The topology and arrows in the neural network structure represent the data flow during prediction, which is different from the data flow during training. Each connection line corresponds to a different weight (the value of which is called a weight), which must be trained.

The operation steps of BPNN are (1) network initialization: give each connection value a random number in the interval (−1, 1), and set the error function *e*, the given calculation accuracy *ε*, and the maximum number of learning times *M*. (2) Randomly select the kth input sample and the corresponding expected output. (3) Calculate the input and output of each neuron in the hidden layer. So, the calculations are shown in

(4) $$\begin{array}{c} hi_{h}\left(k\right)=\sum_{i-1}^{n}w_{ih}xi\left(k\right)-b_{h}, \end{array}$$

(5) $$\begin{array}{c} ho_{h}\left(k\right)=f\left({\text{hi}}_{h}\left(k\right)\right). \end{array}$$

hi_*h*_ is the input vector of the hidden layer; ho_*h*_ is the output vector of the hidden layer; *w*_*ih*_ is the connection weight between the input and the intermediate layer; *b*_*h*_ is the threshold of each neuron in the hidden layer; *f*() is the activation function of the vector.

(6) $$\begin{array}{c} {\text{yi}}_{o}\left(k\right)=\sum_{h=1}^{p}w_{\text{ho}}{\text{ho}}_{h}\left(k\right)-b_{o},\\ {\text{yo}}_{o}\left(k\right)=f\left({\text{yi}}_{o}\left(k\right)\right). \end{array}$$

yi_*o*_ is the input vector of the output layer; yo_*o*_ is the output vector of the output layer; *w*_ho_ is the connection weight between the hidden and the output layer; *b*_*o*_ is the threshold of each neuron in the output layer.

(4) The expected and actual output of the network is used to calculate the partial derivative of the error function concerning each neuron in the output layer.

(5) The partial derivative value of each neuron in the output layer and the input of the hidden layer is used to correct the connection weight, as shown in

(7) $$\begin{array}{c} \Delta w_{\text{ho}}\left(k\right)=-\mu \frac{\partial e}{\partial w_{\text{ho}}} \end{array}$$

(8) $$\begin{array}{c} w_{\text{ho}}^{\left(N+1\right)}=w_{\text{ho}}^{N}+\eta \delta_{o}\left(k\right){\text{ho}}_{h}\left(k\right). \end{array}$$

△*w*_ho_ is the change value of the connection weight; *δ*_*o*_(*k*) is the partial derivative value of each neuron in the output layer.

### 2.5. Street Landscape Planning and Design Based on AI Interactive Experience

Determining the design vision of the streetscape under the intelligent interactive experience is an important preliminary task to support the long-term development of the street. At the beginning of the design, the next feasible and developable design vision or design goal is determined, which can lay a good foundation for the future development of the street. Based on the AI interactive experience, the streetscape is planned and designed. The planning and design process can be divided into two stages, as shown in Figure 5.

In Figure 5, the streetscape vision under the intelligent interactive experience can be planned in two stages. The first part is the short-term design planning vision or design planning goal. The short-term and micro-planning and design visions are to solve practical problems at the current stage, with the main goal of rapidly improving the overall landscape quality of the street and improving the living comfort level of the current street. Typically, this process takes 1–3 years to complete. The main street planning and design vision has 5 points. (1) Create an ideal social place that is fluid, complete, and pleasant; (2) create a pleasant streetscape; (3) create a comfortable, professional, and personalized business office area; (4) provide a new intelligent and intelligent interactive tour experience; (5) show multi-angle, multi-form street features. However, the five short-term micro-design visions may be slightly different in the actual project. The core significance lies in the need to achieve certain design and planning expectations in the short term, improve the overall level of the street in terms of quality, and provide a foundation for the long-term macro planning and design vision.

The streetscape model selects CSiXRevit 2022 software. CSiXRevit 2022 is a very professional architectural modeling software. Additionally, it is also an application plug-in for the “Autodesk Revit” platform. The software has a graphical user interface, various tools are well laid out, and there are powerful modeling capabilities. Rich materials allow for a wider range of modeling.

The long-term street landscape planning and design vision usually has four points: (1) to create the image of the city's core streets; (2) to highlight the urban cultural heritage and regional characteristics; (3) to improve the surrounding economic level; (4) to become the urban street landscape planning and design development benchmarks. CSiXRevit 2022 software simulates the urban streetscape. Meanwhile, AI neural networks are used to analyze the streetscape. The relevant data are entered into the streetscape model. The specific design steps are shown in Figure 6.

In Figure 6, the streetscape planning and design are divided into seven steps. Step 1 is to find information about the location of the street. Step 2 is to conduct on-site research and on-site interviews. Step 3 determines the vision and design goals of the streetscape design. Step 4 proposes the design strategies, principles, and techniques of the streetscape. Step 5 selects the intelligent interactive experience mode. Virtual reality (VR) or intelligent interactive devices are added to the street landscape, and visual landscape immersion techniques or integrated landscape immersion techniques are used to integrate technology and landscape in spiritual and realistic levels in street landscape design. Step 6 carries out specific streetscape planning and design and uses CSiXRevit 2022 to conduct streetscape modeling experiments. Image classification technology integrates intelligent interactive experiences into streetscape models through digital analysis. Step 7 is the implementation of the plan.

### 2.6. Street Landscape Planning Evaluation Based on AI Interactive Experience

AHP and BPNN structures are used to evaluate the effect of streetscape design. Firstly, AHP is used to confirm the evaluation index weights. A total of 100 questionnaires are distributed to passers-by in the relevant streets and the management department staff, and 94 valid questionnaires are recovered. The questionnaire is designed according to the Likert scale, and people's opinions in different fields are aggregated. The mean and standard deviation methods are used to calculate the reasonableness of its indicators. The questionnaires are organized after the feedback of the scores for each indicator. In expert scoring, indicators with lower scores are deleted. Additionally, new indicators are added. Finally, three primary indicators and seven secondary indicators are selected. The AI interactive experience street landscape evaluation index system is shown in Figure 7.

In Figure 7, the streetscape design is evaluated from three perspectives. (1) Street attractiveness is evaluated from three aspects: landscape diversity, landscape characteristics, and infrastructure perfection. (2) Street vitality is evaluated from street air quality and street income. (3) Street carrying capacity is evaluated on pedestrian and resident satisfaction. The calculation weight structure of AHP is shown in Table 1.

In Table 1, the weight of landscape diversity is 0.25; the landscape characteristics is 0.155; the infrastructure perfection is 0.363; the street air quality is 0.195; the street income is 0.325; the pedestrian satisfaction is 0.614; the residents' satisfaction is 0.383.

After the valid questionnaires are sorted and analyzed, the basic information of the respondents is obtained, as shown in Figure 8.

In Figure 8, among the surveyed persons, there are 45 males, 49 females, 54 pedestrians, and 40 residents. The number of people aged 18–22 is 21; aged 22–30 is 25; aged 30–45 is 28; and over 45 is 20.

Statistical Product Service Solutions (SPSS) statistical software is used to analyze the data. Cronbach's alpha coefficient for the survey data is 0.797. Within the scope of the reliability of the questionnaire, the results of the questionnaire are credible.

## 3. Results

### 3.1. Analysis of Factors Affecting the Intelligent Interactive Experience of Streetscape

The respondents' satisfaction with the intelligent interactive streetscape and their preferred intelligent interactive facility survey data are analyzed, as shown in Figure 9.

In Figure 9, in the landscape design, the street night lighting score is 0.832; the overall layout score of the street landscape is 0.795; the street interactive building score is 0.621; the street landscape richness score is 0.532. Therefore, the variety and richness of the streetscape are increased. Additionally, the streets are set up with interactive buildings, such as musical fountains and related artistic buildings. The results showed that the score for the outdoor gallery is 0.532; the score for intelligent garbage classification is 0.326; the score for stair seat is 0.438; the score for LED water light graffiti is 0.651; the score for the interactive music fountain is 0.685. Therefore, the selection of intelligent outdoor interactive facilities should prioritize outdoor interactive music fountains and LED water light graffiti.

### 3.2. AI Interactive Experience-Guided Streetscape Design Assessment

The streetscape design guided by the AI interactive experience is evaluated. According to the weight of each index determined by the questionnaire survey and the AHP, combined with BPNN to calculate, the preoperation result is shown in Figure 10.

In Figure 10, the relative errors of the expected and simulated outputs of the evaluation model after training are 0.016, 0.033, 0.022, 0.019, 0.031, and 0.037, respectively. The relative error results are all lower than 4%, and the error range is reasonable. The simulation evaluation results are the same as the original data results, which can be used to evaluate the design effect of the streetscape comprehensively. The results of the streetscape assessment are shown in Table 2.

In Table 2, the comprehensive evaluation score of the street landscape is 0.60, indicating that the effect of street landscape design is excellent. The comprehensive evaluation values of the three project layers are 0.65, 0.48, and 0.67, respectively. Those data indicate that the carrying capacity index of the street is the best, and the vitality index is the weakest. The environmental condition of the streets is relatively good, but the level of economic development and the comprehensive social conditions still need to be improved. Therefore, when designing the street landscape, the economic development of the street is emphasized, such as attracting investment or introducing large-scale exhibition shops to increase street income. Additionally, the construction of street public facilities has been strengthened, focusing on the street experience of the public, and setting up a Geographic Information Science (GIS) guide system between the street shops to increase the tourist experience.

## 4. Conclusion

This work proposes a streetscape design guided by AI interactive experience and uses AHP and AI technology to evaluate the effect. The results show that (1) the variety and richness of the streetscape should be increased. Additionally, in the street, interactive buildings should be set. (2) The lowest score of street facilities is intelligent garbage classification; the score is 0.326. The interactive music fountain had the highest score of 0.685. (3) The comprehensive evaluation score of the street landscape is 0.60, and the design effect is excellent. The comprehensive evaluation values of the three project layers are 0.65, 0.48, and 0.67, respectively. Those data indicate that the bearing capacity index is the best, and the vitality index is the weakest. Therefore, when designing streetscapes, economic development should be emphasized, such as attracting investment or introducing large-scale exhibition shops to increase street income. Additionally, the construction of street public facilities should be strengthened, and the public street experience should be further emphasized. The survey results can provide a reference for the subsequent design and planning of the streetscape. There are certain deficiencies in the survey data and the influencing factors of intelligent interaction. In the future, the scope of the investigation will be further expanded. A more in-depth investigation of influencing factors will be undertaken. Additionally, big data analysis technology keeps pace with the times, and new technologies will be updated and used in the future. The theory and practice are deeply integrated, and an evaluation model closer to the survey results is designed. The innovation lies in the use of AI technology, which increases the credibility of the experiment.

## Figures and Tables

**Figure 1:** The relationship between intelligent interaction and digital technology, AI, and interaction design.

**Figure 2:** Objects of landscape design for intelligent interactive experience street.

**Figure 3:** AHP. (a) is AHP steps; (b) is the hierarchy of decision goals.

**Figure 4:** BPNN operation structure and operation steps. (a) is BPNN structure; (b) is BPNN operation steps.

**Figure 5:** Streetscape planning: (a) short-term design vision; (b) long-term plan.

**Figure 6:** Setup steps for AI streetscape.

**Figure 7:** Metrics for streetscape assessment.

**Figure 8:** Details of the respondents; (a) identity of the respondents; (b) age distribution of the respondents.

**Figure 9:** Survey results of respondents on intelligent interactive streetscape: (a) satisfaction with intelligent interactive streets; (b) selection results of intelligent interactive facilities.

**Figure 10:** Survey results.

**Table 1:** Weight structure of streetscape assessment indicators.

Index	Weight
Landscape diversity	0.25
Landscape character	0.155
Infrastructure integrity	0.363
Street air quality	0.195
Street income	0.325
Pedestrian satisfaction	0.614
Resident satisfaction	0.383

**Table 2:** Evaluation results.

Synthetic assessment values	0.6
Allure	0.65
Vitality	0.48
Load carrying capacity	0.67

## Data Availability

The authors declare that the data supporting the findings of this study can be obtained from the corresponding author upon request.
